# A Decision Model for the Control and Dissemination of the Online Public Opinions: An Empirical Study of Public Opinion Dissemination on Fraudulent Insurance Claims in Taihe, China

**DOI:** 10.1155/2022/3135149

**Published:** 2022-06-06

**Authors:** Jiangjie Sun, Hui Li, Ning Xu, Zongmin Qiao, Chengsen He

**Affiliations:** ^1^Health Management College, Anhui Medical University, Hefei 230032, China; ^2^Clinical Medical College Anhui Medical University, Hefei 230031, China; ^3^School of Pharmacy, Anhui Medical University, Hefei, Anhui 230032, China; ^4^School of Mathematics and Statistics, Hefei Normal University, Hefei, Anhui 230601, China; ^5^Law College, Anhui Medical University, Hefei 230032, China

## Abstract

This work establishes the SE-IR model of dissemination of online public opinions and control decisions. The model is developed by sorting out the development process of dissemination of the online public opinion model, analysing the mechanism of public opinion evolution in emergencies, drawing on the construction idea of the SEIR contagion model, and combining the characteristics of the online public opinion dissemination with the role mechanism of government intervention. Using this model, we determine the equilibrium point and stability of public opinion dissemination. Using the data of public opinion on an incident of fraudulent insurance claims in China, we explore the influence of different government decisions on public opinion dissemination. The results show that government actions in that case achieved the purpose of minimising the risk of harmful public opinion dissemination.

## 1. Introduction

In the late 1990s, the German sociologist Beck proposed that the development of the social structures has produced huge changes, the traditional era of profit distribution has passed, and the global era of risk allocation has fully arrived [1]. Risk is inevitable, especially after major emergencies, which often trigger a chain reaction, such that the spread of human emotions, attitudes, and opinions may cause group panic or increase social instability. The dissemination of emotions, attitudes, and opinions is referred to as the spread of public opinion [2]. Thus, emergency management is indispensable.

Communications made using modern Internet-based opportunities have revolutionised the way people exchange information, allowing real-time discussions among a huge number of users [3]. The resulting dissemination of public opinions may not only exacerbate the difficulty of handling the original emergency but also trigger new social security incidents. Compared with the public opinions expressed under general events, the public opinions caused by major emergencies gain higher attention and faster transmission speed. Without scientific and reasonable treatment, such opinions could easily trigger mass incidents and then produce secondary disasters. Changes in the public's perception of major emergencies and public opinion lead to differences in their attitudes during the dissemination of public opinions [4].

In this paper, the term *online public opinions* refers to the dissemination of public communication in which netizens express their attitudes, opinions, and emotions towards a certain event, using the Internet as the carrier and the network news media as the platform [5]. Online public opinions about emergencies concern the public social opinion on emergencies reflected by netizens through the Internet, which represents an internet mapping of netizens' public opinion [6]. Major emergencies have a deep social impact and involve a wide range of people.

In addition, with the rapid internet dissemination, improper supervision of the online public opinions and information dissemination will easily trigger negative public sentiment and lead to mass radical behaviours or social instability. For example, the Fukushima nuclear leakage in 2011 triggered a huge buying frenzy of iodised products, such as iodised salt, in the Asia-Pacific region [7]. In 2015, an explosion in Tianjin, China, caused a wave of public opinion due to the “rumours” of disseminators [4], which negatively affected the image of the government's public opinion governance and weakened the government's credibility. At the end of 2020, the insurance fraud events of several hospitals in Taihe County, Anhui Province (referred to as the Taihe Event), achieved a good network public opinion communication effect. In terms of crisis response, the Taihe event met the emergency management requirements of “fast, accurate, and stable” and achieved good results in the aftermath. To a great extent, it reflected the improvement of the government's emergency risk management level.

At present, the risk management literature on online public opinion mainly includes control and theoretical research on secondary disasters caused by public opinions and research on the law of public opinion dissemination and risk management caused by the emergencies themselves. The control and theoretical study of secondary disasters caused by public opinions involves the study of public panic behaviours (such as rush behaviour) caused by emergencies from the perspectives of social psychology, media communication, rumour interference, government control, and public education.

Fan et al. analysed and explained psychobehavioural science as the psychological mechanism of the rush to buy during SARS in China [8], suggesting that the rush to buy was an automatic response stemming from the high level of emotional arousal of the public in a crisis. Lu and Shao used the basic method of system dynamics to construct the analysis process of the snapping system and analysed the causal loop diagram of the snapping event, achieving results showing that the level of public panic is the key intrinsic variable affecting the system of the snapping event [9]. Wei et al. developed a theoretical model of the dynamics of group purchasing behaviour based on group behavioural dynamics theory [10]. They tested this model with a case study of salt purchasing in China triggered by the nuclear crisis in Japan, which showed that individuals' purchasing behaviour was driven by their intrinsic need for life safety and influenced by external group environmental factors. They explained the mechanism of rush behaviour in terms of social psychological or behavioural theories. In 2015, Zhao et al. established a physical model of group purchasing behaviour under emergencies from the perspective of quantitative analysis, attempted to construct a noise heterogeneous opinion propagation model with emergencies as a specific context by using the bounded trust rule approach in opinion dynamics, and analysed the inner law of group opinion evolution in group purchasing behaviour through computer simulation experiments [11].

The research on the communication patterns and risk management of public opinions triggered by emergencies themselves can be broadly divided into two categories: the study of influencing factors and communication process models. Mora et al. studied the cognitive behaviour of people on the seismic safety of buildings after the Canterbury earthquake in the United Kingdom through Twitter and group discussions and found that the design of buildings for life protection was more important than their functional design [12]. Demongeot and Volpert investigated the interaction between individual decisions and external environmental variables (other individuals, public opinions, and some visual and verbal information) [13].

The communication process modelling studies include two categories; the first focuses on the bottom-up modelling approach, such as the evolution of the online public opinions focusing on the interactions between individuals. Representative studies include meta-automata models of opinion propagation [14, 15] and complex system models of opinion propagation dynamics emerging through subject interactions [16, 17]. The strength of these models is that they can better study the state of individual-individual interactions, but their biggest shortcoming is that they cannot simulate the real situation in the real world very well. The other category focuses on the top-down modelling approach and considers the evolution of online opinions of macro groups. The current research findings include the emergent model [18] and the contagion model [19–23]. This model can accurately describe the current situation of changes in public opinion hotspots at each time node, especially the infectious disease model, which is modelled by differential equations and has the rigour of mathematical reasoning. The value of using this mechanism to analyse the law of changes in public opinion and predict the future trend and characteristics of public opinion is highly plastic. In this study, based on the construction mechanism of the infectious disease model, we will explore and propose a derivative model for the control of the online public opinions of major emergencies.

## 2. Presentation of the Model

In 1927, Kermack and McKendrick proposed the classic compartmental model [24]. Let the population size be *N*, divided into susceptible, infected, and removed persons, with the number of people denoted by *S*, *I*, and *R*, respectively, which are all functions of time *t*. The proportion of each part of the population in the overall population is s, *i*, and *r*, which are all functions of time *t*. Let the average number of effective contacts (enough contact to cause transmission) between an individual and others per unit time be *I* and the number of people cured per unit time be *R*. Then, the Susceptible-Infected-Recovered model (SIR Model) can be established:

(1) $$\begin{array}{c} \left\{\begin{array}{c} \frac{dS}{dt}=-\frac{\beta IS}{N},\\ \frac{dI}{dt}=-rI,\\ \frac{dR}{dt}=rI, \end{array}\right. \end{array}$$

and *S* + *I* + *R* = *N*.

The model, despite its simplicity, has been used to study infectious diseases with lifelong immunity after recovery, and it has yielded very valuable concepts and conclusions. In 1985, Sudbury drew on the infectious disease SIR model to study the spread of rumours [19] and obtained that the population size tends to infinity and the proportion of the population that never hears a rumour converges in probability to a limiting constant (approximately 0.203). Zhao et al. combed through the selection behaviour of individuals in the new media era of rumour transmission on the basis of prior studies [25], presenting a modified flow chart of the rumour spreading process with the SIR^∗^ (Susceptible, Infected, and Recovered) model.

(2) $$\begin{array}{c} \left\{\begin{array}{c} \frac{dS}{dt}=-\lambda \overset{¯}{k}\text{IS}-\overset{¯}{k}S\left(\gamma S+\eta R\right)-\delta S,\\ \frac{dI}{dt}=-\overset{¯}{k}\text{IS},\\ \frac{dR}{dt}=\left(1-\lambda \right)\overset{¯}{k}\text{IS}+\overset{¯}{k}S\left(\gamma S+\eta R\right)+\delta S. \end{array}\right. \end{array}$$

Here, $\overset{¯}{k}$ denotes the average degree of the network; *I*, *S*, and *R* denote the density of ignorants, spreaders, and stiflers at time *t*, respectively; and *I* + *S* + *R* = 1. As shown in SIR^∗^, from the spreader's point of view, in time *t*, a spreader spontaneously loses interest in or forgets about a rumour with probability *δ*. Stiflers have a negative effect on a spreader when the spreader tries to disseminate a rumour to a stifler. Suppose that stiflers choose not to propagate a rumour because of disbelief or uninterest; in this case, a spreader turns into a stifler with probability *η* when they contact a stifler. If a spreader contacts another spreader in the rumour spreading process, they may have different versions of the rumour due to individual modification and representation of the rumour. In this situation, the initial spreader may change into a stifler with a probability *γ* because they may doubt the credibility of the rumour. In keeping with reality, *γ* is restricted to be smaller than *η*, i.e., *γ* < *η*.

In 2018, based on the SIR model, Zhang et al. proposed the cross-network communication model SI^3^R for public opinion in coupled networks [21]. The dynamic transfer equations of the SI^3^R model are stated as follows:

(3) $$\begin{array}{c} \left\{\begin{array}{c} \frac{dS}{dt}=A-\alpha_{1}I_{1}S-\alpha_{2}S\left(I_{1}+I_{2}\right)-\alpha_{3}S,\\ \frac{dI_{1}}{dt}=\alpha_{1}I_{1}S-\lambda_{1}I_{1},\\ \frac{dI_{2}}{dt}=\alpha_{2}S\left(I_{1}+I_{2}\right)-\beta I_{2}-\lambda_{2}I_{2},\\ \frac{dI_{3}}{dt}=\beta I_{2}-\lambda_{3}I_{3},\\ \frac{dR}{dt}=\lambda_{1}I_{1}+\lambda_{2}I_{2}+\lambda_{3}I_{3}+\alpha_{3}S. \end{array}\right. \end{array}$$

The model has seven parameters: *λ*_1_, *λ*_1_, *λ*_3_, *α*_1_, *α*_2_, *α*_3_, and *β*, whose connotations are given in Zhang et al.'s paper [21].

The above models argue that the unknowns will inevitably change their state once they are informed of rumours by disseminators. In fact, in reality, in the face of public opinion information, there exists a certain group of people who may not change their status and become lurkers (know the information of the public opinion but are in a state of wandering about whether to spread it, or there is information interaction but they not involved in spreading it). This group is not covered by this model. Because Afassinou considered the differences in the spread of information when individuals receive it, the classical SIR rumour spread model based on the classical SIR rumour spread model was extended to consider the forgetting mechanism and the education rate of the population, resulting in the SEIR rumour spread model [26]. Here, the system of nonlinear ordinary differential equations for the dynamic behaviour of the SEIR rumour propagation model is as follows:

(4) $$\begin{array}{c} \left\{\begin{array}{c} \frac{dS}{dt}=-\lambda \overset{¯}{k}\text{IS}+\lambda_{e}\overset{¯}{k}ES-\alpha \overset{¯}{k}S\left(S+R\right)-\delta \text{S},\\ \frac{dE}{dt}=-\left(\lambda_{e}+\beta_{e}\right)\overset{¯}{k}ES,\\ \frac{dI}{dt}=-\left(\lambda +\beta \right)\overset{¯}{k}\text{IS},\\ \frac{dR}{dt}=\beta \overset{¯}{k}\text{IS}+\beta_{e}\overset{¯}{k}ES+\alpha \overset{¯}{k}S\left(S+R\right)+\delta S, \end{array}\right. \end{array}$$

where $\overset{¯}{k}$ is the average degree of the network. The parameters *λ*, *λ*_*e*_, *β*, and *β*_*e*_ are defined so that 0 ≤ *λ* + *β* ≤ 1 and 0 ≤ *λ*_*e*_ + *β*_*e*_ ≤ 1. The state variables *S*, *E*, *I*, and *R* (all functions of time *t*) are defined so that they obey the normalisation condition: *S* + *E* + *I* + *R* = 1.

In Komi's study, SEIR model analysis is used to determine the final size of rumours and explore the influence of the education rate on the final size of rumours. In 2017, Liu et al. proposed a model of public opinion spreading pattern and control decisions under government intervention for emergencies based on the construction idea of the epidemic SEIR model [27] in the previous study [7]:

(5) $$\begin{array}{c} \left\{\begin{array}{c} \frac{dS}{dt}=\delta -\left(\alpha -\overset{¯}{\alpha }\right)SI-\left(\mu -\overset{¯}{\mu }\right)S,\\ \frac{dE}{dt}=\left(\alpha -\overset{¯}{\alpha }\right)SI-\left(\beta -\overset{¯}{\beta }\right)E-\left(\gamma -\overset{¯}{\gamma }\right)E,\\ \frac{dI}{dt}=\left(\beta -\overset{¯}{\beta }\right)E+\left(\tau -\overset{¯}{\tau }\right)R-\left(\eta -\overset{¯}{\eta }\right)I,\\ \frac{dR}{dt}=\left(\gamma -\overset{¯}{\gamma }\right)E+\left(\eta -\overset{¯}{\eta }\right)I+\left(\mu -\overset{¯}{\mu }\right)S-\left(\tau -\overset{¯}{\tau }\right)R. \end{array}\right. \end{array}$$

*dS*/*dt*, *dE*/*dt*, *dI*/*dt*, and *dR*/*dt* indicate the rate of change in the proportion of the number of unknowns, latents, transmitters, and immune persons, respectively. Parameter *α* is the conversion rate of unknowns to latents, which is also the exposure rate of individual transmitters; *μ* is the conversion rate of unknowns to immunes; *β* is the conversion rate of latents to transmitters; *γ* is the conversion rate from latent to immune; *η* is the conversion rate of transmitters to immunisers; and *τ* is the conversion rate of immunisers to transmitters. Parameters $\overset{¯}{\alpha },\overset{¯}{\beta },\overset{¯}{\gamma },\overset{¯}{\tau },\overset{¯}{\eta },\overset{¯}{\mu }$ reflect the role of government intervention in the process of public opinion dissemination and represent the coefficients of government intervention in the conversion of unknown to latent, unknown to immune, latent to disseminator, latent to immune, disseminator to immune, and immune to disseminator, respectively. Wang's study addressed the equilibrium point and stability of the model. The model strictly refers to the infectious disease model, increases the incubation period, and adds government interventions in each transformation domain to enhance the practical value of the theory, but in reality, the spread of public opinion may not be strictly sequential; there are cases of absolute immunity of public opinion and the knowledge which also affect the type of spread. Based on these actual situations of public opinion dissemination, we propose the following conceptual model of public opinion dissemination paths (Figure 1).

Considering the complexity and uncertainty of practical problems, we propose the following hypotheses:

**Hypothesis 1 .**

The dissemination of public opinion is mainly due to the dissemination of online public opinion.

**Hypothesis 2 .**

The rate of change in the number of people affected by public opinion is proportional to the product of the susceptible and affected populations.

**Hypothesis 3 .**

The change in the proportion of the number of people in each category accurately portrays the respective changes in the number of people, and *dS*/*dt*, *dE*/*dt*, *dI*/*dt*, and *dR*/*dt* represent the rates of change in the proportion of the number of unknowns, latents, transmitters, and immunes, respectively.

**Hypothesis 4 .**

In the conceptual model diagram of public opinion dissemination, *A* denotes the perturbation rate of the number of new netizens. The total (1 + *A*) is divided into four disjoint subclasses: susceptible class *S* (the proportion of internet users with no knowledge of breaking news), latent class *E* (the percentage of netizens who have received information on breaking news and appeared to interact with the platform but did not spread it), infectious class  *I* (the proportion of internet users who have received information about breaking news and have spread public opinions), and removed class  *R* (the proportion of Internet users who have received information about breaking news and have no intention to spread public opinions). Parameters *α*^∗^, *β*^∗^, *ξ*^∗^, *η*^∗^, and *γ*^∗^ all refer to natural transfer factors and *α*^∗^ ∈ [0, 1], *β*^∗^ ∈ [0, 1], *ξ*^∗^ ∈ [0, 1], *η*^∗^ ∈ [0, 1],  and *γ*^∗^ ∈ [0, 1]. Let *ε* denote a direct immuniser and $\overset{¯}{\alpha }$, $\overset{¯}{\beta }$, $\overset{¯}{\eta }$, $\overset{¯}{\xi }$, and $\overset{¯}{\gamma }$ denote the government intervention factors $\left(\overset{¯}{\alpha }\in \left[-1,1\right],\overset{¯}{\beta }\in \left[-1,1\right],\overset{¯}{\eta }\in \left[-1,1\right],\overset{¯}{\xi }\in \left[-1,1\right],\overset{¯}{\gamma }\in \left[-1,1\right]\right)$, such that

(6) $$\begin{array}{c} S+E+I+R=1+A\text{ and }\varepsilon S=\eta^{*}E. \end{array}$$

**Hypothesis 5 .**

$\alpha^{*}-\overset{¯}{\alpha }\in \left[0,1\right]$ ; $\beta^{*}+\overset{¯}{\beta }\in \left[0,1\right]$; $\xi^{*}-\overset{¯}{\xi }\in \left[-1,1\right]$; $\eta^{*}+\overset{¯}{\eta }\in \left[0,1\right]$; $\gamma^{*}-\overset{¯}{\gamma }\in \left[0,1\right]$; and *α* ≥ *ε*.

Based on the above assumptions and the basis of the conceptual model of dissemination of public opinions in emergencies, the current paper proposes the following dynamic equations of the SE-IR model of dissemination of public opinions in major emergencies (Model 1):

(7) $$\begin{array}{c} \left\{\begin{array}{c} \frac{dS}{dt}=A-\left(1-\varepsilon \right)\left(\gamma^{*}-\overset{¯}{\gamma }\right)SI-\left(\alpha^{*}-\overset{¯}{\alpha }\right)S-\varepsilon S,\\ \frac{dE}{dt}=\left(1-\varepsilon \right)\left(\gamma^{*}-\overset{¯}{\gamma }\right)SI-\left(\xi^{*}-\overset{¯}{\xi }+\overset{¯}{\eta }\right)E,\;\\ \frac{dI}{dt}=\left(\alpha^{*}-\overset{¯}{\alpha }\right)S+\left(\xi^{*}-\overset{¯}{\xi }\right)E-\left(\beta^{*}+\overset{¯}{\beta }\right)I,\\ \frac{dR}{dt}=\left(\beta^{*}+\overset{¯}{\beta }\right)I+\left(\eta^{*}+\overset{¯}{\eta }\right)E. \end{array}\right. \end{array}$$

Note that none of the first three equations in Model 1 contains the variable *R*, and *S* + *E* + *I* + *R* = 1 + *A*, and *N* is the total number of internet users at time *t*. Thus, we solve Model 1 by solving only the first three equations of the Model 1. Make the $\alpha =\alpha^{*}-\overset{¯}{\alpha }$, $\beta =\beta^{*}+\overset{¯}{\beta }$, $\xi =\xi^{*}-\overset{¯}{\xi }$, and $\gamma =\gamma^{*}-\overset{¯}{\gamma }$; thus, Model 1 is equivalent to Model 2 and Model 2 is as follows.

(8) $$\begin{array}{c} \left\{\begin{array}{c} \frac{dS}{dt}=A-\left(1-\varepsilon \right)\gamma SI-\left(\alpha +\varepsilon \right)S,\\ \frac{dE}{dt}=\left(1-\varepsilon \right)\gamma SI-\left(\xi +\overset{¯}{\eta }\right)E,\\ \frac{dI}{dt}=\alpha S+\xi E-\beta I. \end{array}\right. \end{array}$$

## 3. Results

According to propagation dynamics theory [28, 29], a threshold exists for any propagation. If  *R*_0_ ≤ 1, then the propagation gradually disappears; if  *R*_0_ > 1, then propagation occurs within a certain range.

**Definition 1 .**

In Model 2, if  *I* = 0, then the model singularity is called the *zero propagation equilibrium point* of SE-IR model 2 for the dissemination of public opinion on major emergencies.

**Theorem 1 .**

The zero propagation equilibrium point for Model 2 is  *P*_0_(*A*/(*α* + *ε*), *εA*/(*η*^∗^(*α* + *ε*)), 0), and if  *R*_0_ ≤ 1, the model is asymptotically stable at *P*_0_.

**Proof**

(Step 1) Prove the existence of a zero propagation equilibrium point.

In Model 2, if the right-hand side of each equation is 0, then,

(9) $$\begin{array}{c} \left\{\begin{array}{c} A-\left(1-\varepsilon \right)\gamma SI-\left(\alpha +\varepsilon \right)S=0,\\ \left(1-\varepsilon \right)\gamma SI-\left(\xi +\overset{¯}{\eta }\right)E=0,\\ \alpha S+\xi E-\beta I=0. \end{array}\right. \end{array}$$

From the definition of zero propagation equilibrium point, *I* = 0, then,

(10) $$\begin{array}{c} \left\{\begin{array}{c} S=\frac{A}{\alpha +\varepsilon },\\ E=\frac{\varepsilon A}{\eta^{*}\left(\alpha +\varepsilon \right)},\\ I=0. \end{array}\right. \end{array}$$

(Step 2) Find the zero-point threshold *R*_0_ for Model 2.

Letting

(11) $$\begin{array}{c} T=\left(\begin{array}{c} E\\ I\\ S \end{array}\right), \end{array}$$

Model 2 can be simplified to $dT/dt=\tilde{F}\left(t\right)-\tilde{V}\left(t\right)$, where $\tilde{F}\left(t\right)$ denotes the rate of increase of nascent variables and $\tilde{V}\left(t\right)$ denotes the population intergroup transfer rate. Then, we have

(12) $$\begin{array}{c} \tilde{F}\left(t\right)=\left(\begin{array}{c} \left(1-\varepsilon \right)\gamma SI\\ 0\\ 0 \end{array}\right)\text{and }\tilde{V}\left(t\right)=\left(\begin{array}{c} \left(\xi +\overset{¯}{\eta }\right)E\\ \;\beta I-\xi E-\alpha S\\ \left(1-\varepsilon \right)\gamma SI+\left(\alpha +\varepsilon \right)S-A \end{array}\right). \end{array}$$

Since the spread of public opinions is only related to the rate of change of *E* and *I*, we calculate the Jacobi matrices corresponding to $\tilde{F}\left(t\right)$ and $\tilde{V}\left(t\right)$ with respect to the variables *E* and *I*, denoted as *F*(*t*) and *V*(*t*), respectively. Then, we have

(13) $$\begin{array}{c} {\left.F\left(t\right)\right|}_{I=0}=\left(\begin{array}{cc} \frac{\partial F_{1}}{\partial E} & \frac{\partial F_{1}}{\partial I}\\ \frac{\partial F_{2}}{\partial E} & \frac{\partial F_{2}}{\partial I} \end{array}\right)=\left(\begin{array}{cc} 0 & \left(1-\varepsilon \right)\gamma S\\ 0 & 0 \end{array}\right), \end{array}$$

(14) $$\begin{array}{c} {\left.V\left(t\right)\right|}_{I=0}=\left(\begin{array}{cc} \frac{\partial V_{1}}{\partial E} & \frac{\partial V_{1}}{\partial I}\\ \frac{\partial V_{2}}{\partial E} & \frac{\partial V_{2}}{\partial I} \end{array}\right)=\left(\begin{array}{cc} \xi +\overset{¯}{\eta } & 0\\ -\xi & \beta \end{array}\right)=\left(\begin{array}{cc} \overset{¯}{\eta } & 0\\ 0 & \beta \end{array}\right). \end{array}$$

Further, we find that

(15) $$\begin{array}{c} {\left.V^{-1}\left(t\right)\right|}_{I=0}=\left(\begin{array}{cc} \frac{1}{\overset{¯}{\eta }} & 0\\ 0 & \frac{1}{\beta } \end{array}\right), \end{array}$$

so there is a regeneration matrix

(16) $$\begin{array}{c} F\left(t\right){\left|{}_{I=0}\times V^{-1}\left(t\right)\right|}_{I=0}=\left(\begin{array}{cc} 0 & \frac{\left(1-\varepsilon \right)\gamma S}{\beta }\\ 0 & 0 \end{array}\right). \end{array}$$

Based on the results of Driessche and Watmough, the spectral radius of the regeneration matrix can be obtained [30]:

(17) $$\begin{array}{c} R_{0}=\rho \left(F\left(t\right){\left|{}_{I=0}\times V^{-1}\left(t\right)\right|}_{I=0}\right)=\underset{1\leq i\leq 2}{\max}\left|\lambda_{i}\right|=\frac{\left(1-\varepsilon \right)\gamma S}{\beta }=\frac{\left(1-\varepsilon \right)\gamma A}{\beta \left(\alpha +\varepsilon \right)}. \end{array}$$

(Step 3) If  *R*_0_ ≤ 1, Model 2 is asymptotically stable at zero equilibrium *P*_0_

In Model 2, if the right side of each equation is *X*, *Y*, and *Z*

(18) $$\begin{array}{c} \left\{\begin{array}{c} X=A-\left(1-\varepsilon \right)\gamma SI-\left(\alpha +\varepsilon \right)S,\\ Y=\left(1-\varepsilon \right)\gamma SI-\left(\xi +\overset{¯}{\eta }\right)E,\\ Z=\alpha S+\xi E-\beta I. \end{array}\right. \end{array}$$

Then, the Jacobian matrix of system (18) is

(19) $$\begin{array}{c} \text{J}=\left(\begin{array}{ccc} \frac{\partial X}{\partial S} & \frac{\partial X}{\partial E} & \frac{\partial X}{\partial I}\\ \frac{\partial Y}{\partial S} & \frac{\partial Y}{\partial E} & \frac{\partial Y}{\partial I}\\ \frac{\partial Z}{\partial S} & \frac{\partial Z}{\partial E} & \frac{\partial Z}{\partial I} \end{array}\right)=\left(\begin{array}{ccc} -\left(1-\varepsilon \right)\gamma I-\left(\alpha +\varepsilon \right) & 0 & -\left(1-\varepsilon \right)\gamma S\\ \left(1-\varepsilon \right)\gamma I & -\left(\xi +\overset{¯}{\eta }\right) & \left(1-\varepsilon \right)\gamma S\\ \alpha & \xi & -\beta \end{array}\right). \end{array}$$

Thus, the results are as follows:

(20) $$\begin{array}{c} J\left(P_{0}\right)=J\left(\frac{A}{\alpha +\varepsilon },\frac{\varepsilon A}{\eta^{*}\left(\alpha +\varepsilon \right)},0\right)=\left(\begin{array}{ccc} -\varepsilon & 0 & -\frac{\left(1-\varepsilon \right)\gamma A}{\varepsilon }\\ 0 & -\overset{¯}{\eta } & \frac{\left(1-\varepsilon \right)\gamma A}{\varepsilon }\\ 0 & 0 & -\beta \end{array}\right). \end{array}$$

Then, its corresponding characteristic equation is as follows:

(21) $$\begin{array}{c} \left(J\left(P_{0}\right)-\lambda E\right)X=0. \end{array}$$

The sufficient and necessary conditions for it to have a nonzero solution are as follows:

(22) $$\begin{array}{c} \left|J\left(P_{0}\right)-\lambda E\right|=0. \end{array}$$

Then,

(23) $$\begin{array}{c} \left|\begin{array}{ccc} -\lambda -\varepsilon & 0 & -\frac{\left(1-\varepsilon \right)\gamma A}{\varepsilon }\\ 0 & -\lambda -\overset{¯}{\eta } & \frac{\left(1-\varepsilon \right)\gamma A}{\varepsilon }\\ 0 & 0 & -\lambda -\beta \end{array}\right|=0. \end{array}$$

Then,

(24) $$\begin{array}{c} \left[-\lambda -\varepsilon \right]\times \left(-\lambda -\overset{¯}{\eta }\right)\times \left(-\lambda -\beta \right)=0. \end{array}$$

Thus, the roots of system (22) are all negative. That is, if *R*_0_ ≤1, then Model 2 is asymptotically stable at *P*_0_ [31, 32]. In particular, if *ε* = 0, our results are consistent with those of previous studies [7, 33].

**Theorem 2 .**

There exists a nonzero propagation equilibrium point for Model 2 as

(25) $$\begin{array}{c} P_{*}\left(\frac{A\eta^{*}}{\varepsilon \left(\xi +\eta^{*}\right)+\varepsilon \overset{¯}{\eta }+\alpha \eta^{*}},\frac{\varepsilon A}{\varepsilon \left(\xi +\eta^{*}\right)+\varepsilon \overset{¯}{\eta }+\alpha \eta^{*}},\frac{\left(\alpha \beta \eta^{*}+\alpha \xi \right)A}{\beta \left[\varepsilon \left(\xi +\eta^{*}\right)+\varepsilon \overset{¯}{\eta }+\alpha \eta^{*}\right]}\right), \end{array}$$

and if  *R*_0_ >1, then the model is locally asymptotically stable at *P*_∗_.

**Proof**

(Step 1) Prove the existence of a zero propagation equilibrium point.

In Model 2, if the right-hand side of each equation is 0, then,

(26) $$\begin{array}{c} \left\{\begin{array}{c} A-\left(1-\varepsilon \right)\gamma SI-\left(\alpha +\varepsilon \right)S=0,\\ \left(1-\varepsilon \right)\gamma SI-\left(\xi +\overset{¯}{\eta }\right)E=0,\\ \alpha S+\xi E-\beta I=0. \end{array}\right. \end{array}$$

The first and second equations in system (26) are added together and combined with equation *εS* = *η*^∗^*E* to form the system of

(27) $$\begin{array}{c} \left\{\begin{array}{c} A-\left(\xi +\overset{¯}{\eta }\right)E-\left(\alpha +\varepsilon \right)S=0,\\ \alpha S+\xi E-\beta I=0,\\ \varepsilon S=\eta^{*}E. \end{array}\right. \end{array}$$

The third equation of system (27) yields *E*, the second equation yields *I*, and the first equation yields *E* and *I* as follows:

(28) $$\begin{array}{c} \left\{\begin{array}{c} S=\frac{A\eta^{*}}{\varepsilon \left(\xi +\eta^{*}\right)+\varepsilon \overset{¯}{\eta }+\alpha \eta^{*}},\\ E=\frac{\varepsilon A}{\varepsilon \left(\xi +\eta^{*}\right)+\varepsilon \overset{¯}{\eta }+\alpha \eta^{*}},\\ I=\frac{\left(\alpha \beta \eta^{*}+\alpha \xi \right)A}{\beta \left[\varepsilon \left(\xi +\eta^{*}\right)+\varepsilon \overset{¯}{\eta }+\alpha \eta^{*}\right]}. \end{array}\right. \end{array}$$

(Step 2) Calculate the nonzero threshold *P*_∗_ of Model 2.

The Jacobian matrix corresponding to $\tilde{F}\left(t\right)$ and $\tilde{V}\left(t\right)$ with respect to *E* and *I* variables can be obtained as in Theorem 2.

(29) $$\begin{array}{c} F\left(t\right)=\left(\begin{array}{cc} \frac{\partial F_{1}}{\partial E} & \frac{\partial F_{1}}{\partial I}\\ \frac{\partial F_{2}}{\partial E} & \frac{\partial F_{2}}{\partial I} \end{array}\right)=\left(\begin{array}{cc} 0 & \left(1-\varepsilon \right)\gamma S\\ 0 & 0 \end{array}\right),\\ V\left(t\right)=\left(\begin{array}{cc} \frac{\partial V_{1}}{\partial E} & \frac{\partial V_{1}}{\partial I}\\ \frac{\partial V_{2}}{\partial E} & \frac{\partial V_{2}}{\partial I} \end{array}\right)=\left(\begin{array}{cc} \xi +\overset{¯}{\eta } & 0\\ -\xi & \beta \end{array}\right). \end{array}$$

The following results are obtained

(30) $$\begin{array}{c} V^{-1}\left(t\right)=\left(\begin{array}{cc} \frac{\beta }{\beta \left(\xi +\overset{¯}{\eta }\right)} & \frac{0}{\beta \left(\xi +\overset{¯}{\eta }\right)}\\ -\frac{\xi }{\beta \left(\xi +\overset{¯}{\eta }\right)} & \frac{\xi +\overset{¯}{\eta }}{\beta \left(\xi +\overset{¯}{\eta }\right)} \end{array}\right)=\left(\begin{array}{cc} \frac{1}{\xi +\overset{¯}{\eta }} & 0\\ -\frac{\xi }{\beta \left(\xi +\overset{¯}{\eta }\right)} & \frac{1}{\beta } \end{array}\right). \end{array}$$

Then, the next generation matrix is

(31) $$\begin{array}{c} F\left(t\right)\times V^{-1}\left(t\right)=\left(\begin{array}{cc} -\frac{\xi \left(1-\varepsilon \right)\gamma S}{\beta \left(\xi +\overset{¯}{\eta }\right)} & \frac{\left(1-\varepsilon \right)\gamma S}{\beta }\\ 0 & 0 \end{array}\right). \end{array}$$

Based on the results of Driessche and Watmough, the spectral radius of the next generation matrix can be obtained [30]:

(32) $$\begin{array}{c} R_{0}=\rho \left(F\left(t\right)\times V^{-1}\left(t\right)\right)=\underset{1\leq i\leq 2}{\max}\left|\lambda_{i}\right|=\frac{\xi \left(1-\varepsilon \right)\gamma S}{\beta \left(\xi +\overset{¯}{\eta }\right)}. \end{array}$$

That is,

(33) $$\begin{array}{c} R_{0}=\frac{\xi \left(1-\varepsilon \right)\gamma }{\beta \left(\xi +\overset{¯}{\eta }\right)}\times \frac{A\eta^{*}}{\varepsilon \left(\xi +\eta^{*}\right)+\varepsilon \overset{¯}{\eta }+\alpha \eta^{*}}. \end{array}$$

(Step 3) Show that Model 2 is locally asymptotically stable at the nonzero point *P*_∗_ when  *R*_0_ > 1.

In Model 2, let the right-hand side of each equation be  *X*, *Y*, *Z*, respectively. Then, it follows that

(34) $$\begin{array}{c} \left\{\begin{array}{c} X=A-\left(1-\varepsilon \right)\gamma SI-\left(\alpha +\varepsilon \right)S,\\ Y=\left(1-\varepsilon \right)\gamma SI-\left(\xi +\overset{¯}{\eta }\right)E,\\ Z=\alpha S+\xi E-\beta I. \end{array}\right. \end{array}$$

Then, the Jacobian matrix for system (34) is

(35) $$\begin{array}{c} \text{J}=\left(\begin{array}{ccc} \frac{\partial X}{\partial S} & \frac{\partial X}{\partial E} & \frac{\partial X}{\partial I}\\ \frac{\partial Y}{\partial S} & \frac{\partial Y}{\partial E} & \frac{\partial Y}{\partial I}\\ \frac{\partial Z}{\partial S} & \frac{\partial Z}{\partial E} & \frac{\partial Z}{\partial I} \end{array}\right)=\left(\begin{array}{ccc} -\left(1-\varepsilon \right)\gamma I-\left(\alpha +\varepsilon \right) & 0 & -\left(1-\varepsilon \right)\gamma S\\ \left(1-\varepsilon \right)\gamma I & -\left(\xi +\overset{¯}{\eta }\right) & \left(1-\varepsilon \right)\gamma S\\ \alpha & \xi & -\beta \end{array}\right). \end{array}$$

In summary, the results are as follows

(36) $$\begin{array}{c} J\left(P_{*}\right)=J\left(\frac{A\eta^{*}}{\varepsilon \left(\xi +\eta^{*}\right)+\varepsilon \overset{¯}{\eta }+\alpha \eta^{*}},\frac{\varepsilon A}{\varepsilon \left(\xi +\eta^{*}\right)+\varepsilon \overset{¯}{\eta }+\alpha \eta^{*}},\frac{\left(\alpha \beta \eta^{*}+\alpha \xi \right)A}{\beta \left[\varepsilon \left(\xi +\eta^{*}\right)+\varepsilon \overset{¯}{\eta }+\alpha \eta^{*}\right]}\right). \end{array}$$

If we denote

(37) $$\begin{array}{c} P≜\left(1-\varepsilon \right)\gamma \times \frac{A\eta^{*}}{\varepsilon \left(\xi +\eta^{*}\right)+\varepsilon \overset{¯}{\eta }+\alpha \eta^{*}},\\ Q≜\left(1-\varepsilon \right)\gamma \times \frac{\left(\alpha \beta \eta^{*}+\alpha \xi \right)A}{\beta \left[\varepsilon \left(\xi +\eta^{*}\right)+\varepsilon \overset{¯}{\eta }+\alpha \eta^{*}\right]}. \end{array}$$

Then,

(38) $$\begin{array}{c} 0\leq Q\leq P. \end{array}$$

That is,

(39) $$\begin{array}{c} J\left(P_{*}\right)=\left(\begin{array}{ccc} -Q-\left(\alpha +\varepsilon \right) & 0 & -P\\ \text{Q} & -\left(\xi +\overset{¯}{\eta }\right) & P\\ \alpha & \xi & -\beta \end{array}\right). \end{array}$$

Then, the corresponding characteristic equation is:

(40) $$\begin{array}{c} \left(J\left(P_{*}\right)-\lambda E\right)X=0. \end{array}$$

A sufficient requisite for it to have a nonzero solution is

(41) $$\begin{array}{c} \left|J\left(P_{*}\right)-\lambda E\right|=0. \end{array}$$

Then,

(42) $$\begin{array}{c} \left|\begin{array}{ccc} -Q-\left(\alpha +\varepsilon \right)-\lambda & 0 & -P\\ Q & -\lambda -\left(\xi +\overset{¯}{\eta }\right) & P\\ \alpha & \xi & -\lambda -\beta \end{array}\right|=0. \end{array}$$

That is,

(43) $$\begin{array}{c} \lambda^{3}+a_{1}\lambda^{2}+a_{2}\lambda +a_{3}=0, \end{array}$$

where

(44) $$\begin{array}{c} a_{1}=Q+\alpha +\varepsilon +\beta +\xi +\overset{¯}{\eta },\\ a_{2}=\beta \left(\xi +\overset{¯}{\eta }\right)+\left(\beta +\xi +\overset{¯}{\eta }\right)\left(Q+\alpha +\varepsilon \right)+P\left(\xi -\alpha \right),\\ a_{3}=P\left(\xi \varepsilon -\alpha \overset{¯}{\eta }\right)+\beta \left(\xi +\overset{¯}{\eta }\right)\left(Q+\alpha +\varepsilon \right). \end{array}$$

Because 0 ≤ *Q* ≤ *P*, if *R*_0_ > 1, we have *a*_1_ > 0, *a*_2_ > 0, *a*_3_ > 0, and *a*_1_*a*_2_ − *a*_3_ > 0. It follows from the Routh-Hurwitz discriminant that Model 2 is locally asymptotically stable at the nonzero point *P*_∗_ [34, 35].

## 4. Empirical Analysis

### 4.1. Case Study and Problem Description

On December 14, 2020, Xinjing News first exclusively published the article “Anhui Taihe hospitals suspected of fraudulent insurance: no disease ‘brain infarction,' someone received free hospitalisation 9 times in a year,” which shocked the national medical community. At 15:35 on that day, the Taihe County Medical Insurance Bureau announced that a joint investigation team was set up to investigate. On December 15, 2020, at 02:39, Xinjing News posted the original article, then 2,800 people short comment or retweeted (i.e., posted a short comment article referring to it) and their comments. The National Health Insurance Bureau announced on the 15th that “a working group has been dispatched to supervise in the field and carry out emergency disposal work.” On December 20, Xinjing News posted an article, “8 people detained for suspected insurance fraud at several hospitals in Taihe County: Hospital director detained by the Discipline Inspection Commission for investigation,” and public opinion concerns then dropped back significantly. This drop is enough to show that the work of the administration of the Medicare fund supervision in this public opinion deescalation was successful.

### 4.2. Model Theory Analysis

According to Wang's parameter processing method for public opinion dissemination (Wang, 2017), this study uses

(45) $$\begin{array}{c} R_{0}=\frac{\xi \left(1-\varepsilon \right)\gamma }{\beta \left(\xi +\overset{¯}{\eta }\right)}\times \frac{A\eta^{*}}{\varepsilon \left(\xi +\eta^{*}\right)+\varepsilon \overset{¯}{\eta }+\alpha \eta^{*}}. \end{array}$$

Using the data from the Taihe event, it is possible to obtain *R*_0_ as an inverse proportional function to *ε*; the approximate image is as follows (Figure 2).

Thus, the higher the rate of direct immunisation, the less likely it is that public opinions will be spread. Therefore, according to Afassinou's study, “the dissemination of information when individuals receive it is significantly related to the education rate of the population” [26]. We can improve the education level of social groups to increase the direct immunity rate of the public to public opinions.

### 4.3. Fitting Simulation

Drawing on Wang and Li's parameter processing method of public opinion dissemination [7], we propose the baseline data and hypothetical contextual data shown in Table 1, considering the current state of public opinion dissemination for the Taihe event that occurred in Fuyang, China, in the year 2020 (public opinion data from Xinjing News from December 14-20, 2020).

Based on the above parameters, the degree to which *I* is influenced by each parameter can be obtained as shown below.

In Figure 3, the government's moderating effect on public opinion control is obvious, and the positive effectiveness is much more significant than the negative effectiveness, which is basically consistent with the government's attitude toward public opinion disposal. When the Taihe event was first exposed in Xinjing News on December 14, 2020, the Taihe Medical Insurance Bureau and the county government immediately set up a joint investigation group to investigate the issues reflected by the media, and they released word of the government's intervention through the “Taihe Release” platform at 15:35 on December 14, 2020, which to a certain extent realised the government's role in regulating public opinions.

Combining Figures 3 and 4, we see that the government's regulation of opinion disseminators is significantly lower than that of susceptibles. The government's risk of opinion regulation at this stage is higher, which coincides with the theory of in-the-moment disposal of public opinion control, which requires the timely release of the truth about public opinion events. The risk of further spread of harmful public opinions is great when there is information concealment.

Figure 5 shows that the government's regulating effect on public opinion control is better in the stage of the potential infected transfer, and the positive effect is more significant than the negative effect, which is consistent with the government's attitude toward the disposal of public opinions. On December 15, 2020, the public opinions of the Taihe incident fermented, with more than 2,800 retweets and give a like, 4,800 give a like, 642 retweets, and 642 retweeted,. Attracting 835 short comments after its reporting of the incident, Xinjing News pushed the situation to the climax, and the role of progovernment public opinion regulation was huge in terms of the area involved. Immediately after that, the government of Taihe responded that a joint investigation group had been set up locally and promptly announced that the joint investigation group was composed of the Discipline Inspection Committee, Public Security, Medical Insurance, Health Care, Audit department, and other departments. This information was released in a timely manner and directly stabilised the hearts of the people. Prompted by the Xinjing News on December 20, 2020, the media reported “Taihe County, a number of hospitals suspected of fraudulent insurance, 8 people detained, hospital director detained by the Discipline Inspection Commission for investigation.” After that, concern stabilised, with only 22 retweets, 101 compliments, and 30 comments; the information in those mostly praises the government response as timely and efficient, along with other positive evaluation.

As shown in Figure 6, the government's regulation of public opinion disseminators is significantly lower than that of susceptibles. The government's risk of regulating public opinions at this stage is higher, which coincides with the theory of in-the-moment public opinion control, which requires the timely release of the truth about public opinion events. The risk arising from public opinion is great when information is concealed.

From Figure 7, it can be seen that the timely release of public opinions by the government can effectively increase the direct immunity rate of susceptibles. This stage is also the best time for the government to regulate public opinions, which coincides with the theory of disposing of public opinions in the middle of the matter for optimal public opinion control.

In summary, we see that the government interventions to control public opinion related to the Taihe event were basically in line with the scientific emergency response principles, and the risk control was effective.

## 5. Conclusion

This work considers the effectiveness of the governmental opinion control in the Taihe event, combined with the simulation results of the public opinion dissemination model proposed in this study. The resulting analysis is sufficient to show that the government's public opinion deescalation efforts were successful. The study of this model further suggests that the size of the spectral radius *R*_0_ can determine the public opinion propagation dynamics. The public opinion dissemination model proposed in this study has a unique nonzero propagation equilibrium point, and the model is valid. The study results provide a theoretical basis for establishing public opinion guidance mechanisms and the implementation of effective deescalation measures in response to public opinion during emergencies. To better guide and diffuse public opinion on emergencies, we suggest that the government should establish a regular mechanism for guiding public opinion on emergencies, promptly start emergency response, and respond to public concerns in a timely manner to avoid secondary disasters. At the same time, the government can achieve the overall improvement of working network literacy by enhancing the education level of the public and then enhancing the direct immunity rate of internet users to network public opinion in order to ultimately reduce the risk of harmful network public opinions.

## Figures and Tables

**Figure 1:** Conceptual model of public opinion communication.

**Figure 2:** Plot of spectral radius *R*_0_ versus *ε*.

**Figure 3:** *I* influenced by $\overset{¯}{\alpha }$.

**Figure 4:** *I* influenced by $\overset{¯}{\beta }$.

**Figure 5:** *I* influenced by $\overset{¯}{\xi }$.

**Figure 6:** *I* influenced by $\overset{¯}{\eta }$.

**Figure 7:** *I* influenced by *ε*.

**Table 1:** Value settings for each contextual parameter.

Situations	*A*	*α* ^∗^	$\overset{¯}{\alpha }$	*β* ^∗^	$\overset{¯}{\beta }$	*ξ* ^∗^	$\overset{¯}{\xi }$	*η* ^∗^	$\overset{¯}{\eta }$	*ε*
Baseline	0.02	0.02	0	0.03	0	0.05	0	0.03	0	0.02
Case 1	0.02	0.02	Variable	0.03	0	0.05	0	0.03	0	0.02
Case 2	0.02	0.02	0	0.03	Variable	0.05	0	0.03	0	0.02
Case 3	0.02	0.02	0	0.03	0	0.05	Variable	0.03	0	0.02
Case 4	0.02	0.02	0	0.03	0	0.05	0	0.03	Variable	0.02
Case 5	0.02	0.02	0	0.03	0	0.05	0	0.03	0	Variable

## Data Availability

The data used to support the findings of this study are included within the article.
